The article "Effect of FLOT2 Gene Expression on Invasion and Metastasis of Colorectal Cancer and Its Molecular Mechanism under Nanotechnology and RNA Interference" was retracted in 2024. Reasons: signs of a paper mill; suspected computer-generated content; unreliable results or conclusions; concerns about the data.

# Effect of FLOT2 Gene Expression on Invasion and Metastasis of Colorectal Cancer and Its Molecular Mechanism under Nanotechnology and RNA Interference

**DOI:** 10.1155/2022/2897338

**Published:** 2022-04-04

**Authors:** Chonghan Zhong, Fangfang Zheng, Shanping Ye, Gengmei Gao, Penghui He, Dongning Liu

**Affiliations:** ^1^Department of Gastrointestinal Surgery, The First Affiliated Hospital of Nanchang University, Nanchang 330006, China; ^2^Second Department of Cardiology, The Third Hospital of Nanchang, Nanchang 330009, China

## Abstract

The study is aimed at investigating the effect of the FLOT2 gene on invasion and metastasis of colorectal cancer (CRC) cells and the corresponding molecular mechanism by preparing polylysine-silicon nanoparticles. Specifically, polylysine was used to modify the silica nanoparticles prepared by the emulsification method to obtain polylysine-silicon nanoparticles. The characterization of polylysine-silicon nanoparticles was completed by nanoparticle size analyzer, laser particle size potentiometer, and transmission microscope. The influence of polylysine-silicon nanoparticles on the survival rate of CRC cell line HT-29 was detected using the method of 3-(4,5-dimethylthiazol-2-yl)-2, 5-diphenyltetrazolium bromide (MTT). The FLOT2-siRNA expression vector was constructed and transfected with HT-29. The HT-29 transfected with empty plasmid was used as the negative control (NC). Western Blot (WB) and reverse transcription-polymerase chain reaction (RT-PCR) were used to detect expression levels of FLOT2 gene and epithelial-mesenchymal transition- (EMT-) related genes. Transwell invasion assay, Transwell migration assay, and CCK8 assay were used to detect the cell invasion, migration, and proliferation. The results showed that the average particle size of polylysine-silicon nanoparticles was 30 nm, the potential was 19.65 mV, the particle size was 65.8 nm, and the dispersion coefficient was 0.103. At the same concentration, the toxicity of silicon nanoparticles to HT-29 was significantly lower than that of liposome reagent, and the transfection efficiency was 60%, higher than that of liposome reagent (40%). The mRNA level and protein expression of the FLOT2 gene in the FLOT2-siRNA group were significantly lower than those in the NC group (*P* < 0.01). The optical density (OD) value of the NC group and the blank control (CK) group were significantly higher than that of FLOT2-siRNA cells (*P* < 0.01). The OD value of FLOT2-siRNA cells was lower than that of NC cells at 48 h, 72 h, and 96 h (*P* < 0.01). The mRNA levels and protein expressions of MMP2 and vimentin in the FLOT2-siRNA group were significantly lower than those in the NC group and CK group (*P* < 0.01). The mRNA level and protein expression of the E-cadherin gene in the FLOT2-siRNA group were significantly higher than those in the NC group and CK group (*P* < 0.01). In conclusion, an RNA interference plasmid with high transfection efficiency and low cytotoxicity was established based on nanotechnology. siRNA-mediated FLOT2 protein inhibits the invasion, migration, and proliferation of CRC cells by regulating the expression changes of EMT-related genes, which provides a scientific basis for clinical treatment of CRC.

## 1. Introduction

As a targeted technology, RNA interference plays a key role in gene function verification, immune disease pathogenesis research, and prevention of infectious diseases [1]. The transfection systems commonly used in traditional RNA interference technology mainly include virus vector-mediated system and nonvirus-mediated DNA plasmid vector. Of them, the RNA interference transfection efficiency of virus vector-mediated system is high, but there is still a phenomenon of a small amount of virus protein expression after infection of target cells, which leads to the body's specific immune response. Moreover, vector assembly of the viral vector-mediated RNA interference system is difficult and costly [2]. A nonviral vector is obviously safer and more reliable than the viral vector, but it has the defects of low transfection efficiency and even ineffective expression of target genes when transfecting cells [3]. It is found that traditional RNA interference technologies all have the problem of gene vector selection, and a safe and effective gene vector is the key to the application of gene therapy in clinical treatment. The ideal gene vector should have the advantages of nontoxicity, high efficiency, good targeting, easy preparation, and low price. Therefore, it is of great significance to seek nontoxic gene vectors with high transfection efficiency, simple preparation, and low price. The development of nanotechnology provides new opportunities for the application of RNA interference technology. A nanoparticle-based gene carrier system has the characteristics of safety, high efficiency, and good biocompatibility, and thus, it becomes a new gene carrier [4]. Silicon is a low-toxicity biocompatible nanogene carrier material with easy surface modification. Silicon nanoparticles have been found to be a promising new gene carrier with good cell uptake effect. However, silicon nanoparticles alone cannot mediate DNA transfer, and their surface must be modified by ions or positive groups before they can be used as gene carriers [5]. Strongly positive poly-L-lysine-modified silicon nanoparticles can shield high-density positive charge, thus reducing the cytotoxicity, which has the advantages of good biocompatibility, noncytotoxicity, and easy surface modification, making it possible to become a good gene carrier [6].

Colorectal cancer (CRC) is one of the common malignant tumors of the digestive tract. According to related statistics, the incidence and mortality of CRC ranks the third among digestive tract tumors [7]. The onset of CRC is insidious, and most of the patients are in the middle or late stage when they go to see the doctor. About 55% of the patients have had distant metastases at the time of diagnosis. Although the current methods of surgery, radiotherapy, and chemotherapy have reduced the overall mortality of CRC, the prognostic effect of patients with local and remote metastasis is still not ideal. The current research results believe that invasion and metastasis are the main causes of death in CRC patients [8]. FLOT2 is highly expressed in a variety of tumor tissues and has an obvious correlation with the occurrence and development of tumors [9]. Moreover, FLOT2 expression is positively correlated with the tumor stage and lymphatic metastasis, and it is found that the proliferation of kidney cancer and breast cancer cells can be effectively inhibited after interference with FLOT2 gene [10]; in addition, FLOT2 gene expression is closely related to the invasion and metastasis of gastric cancer [11]. Studies have shown that the decrease of the expression level of FLOT2 protein mediated by siRNA can obviously inhibit the activity of Src tyrosine kinase, thus slowing down the epithelial-mesenchymal transition (EMT) process of human nasopharyngeal carcinoma cell line induced by TGF-*β* [12]. FLOT2 siRNA can reduce the growth and invasion of esophageal squamous cell carcinoma [13]. siRNA-mediated downregulation of FLOT2 expression can inhibit the proliferation, invasion, and migration of gastric cancer cells [14]. Meanwhile, studies have shown that FLOT2 can inhibit the proliferation of breast cancer cells by regulating Akt/FOXO signal transduction and that FLOT2 deficiency can lead to reduced cell metastasis in mouse breast cancer models [15]. These results indicate that the expression of FLOT2 gene is associated with invasion and metastasis of various tumors and is related to the activation of EMT, NF-*κ*B, and Akt/FOXO signaling pathways. CRC metastasis is a very complex process involving multiple factors and steps, in which multiple signal transduction pathways are cross-linked and interact with each other. However, there are few studies on the effect of FLOT2 gene expression on the invasion and metastasis of CRC, and the mechanism is still unclear.

In summary, silicon nanoparticle modified with PLL is a DNA transfection carrier with high biological safety and high TE. There are few studies on the correlation between FLOT2 gene expression and CRC cell invasion and metastasis. In this study, an interference carrier of FLOT2 was constructed with RNA interference technology to explore the expression of siRNA carried by PLL-modified silicon nanoparticles in CRC cells, so as to explore the influence of FLOT2 gene on the invasion and metastasis of CRC and its corresponding molecular mechanism and provide a certain scientific basis for the clinical treatment and prognosis analysis of CRC.

## 2. Materials and Methods

### 2.1. Preparation of Silicon Nanoparticles and Modification of Polylysine

Similar to the hydrolysis method of ethyl orthosilicate in a water-in-oil microemulsion system, the silica nanoparticles were prepared by the emulsification method. The specific operation method was given as follows. After 4.0 g of nonylphenol polyoxyethylene ether, 50 mL of cyclohexane, and 0.6 mL of double distilled water were mixed and stirred completely, hexyl alcohol was added in dropwise to form a stable water/oil (W/O) microemulsion system; ethyl orthosilicate and an appropriate amount of ammonia were added and then stirred at the room temperature for 24 hours; after an appropriate amount of acetone was added, the mixture was centrifuged at 12,000 rpm/min for around 10 minutes to collect the sediment; the sediment was freeze-dried in a freeze drier, grinded into powder, added with 1.0 mL of Na_2_CO_3_ solution, sonicated for 15 minutes on an ice-water bath, and then centrifuged at 12,000 rpm/min for another 10 minutes to collect the sediment again; a 1.0 mL of resuspension liquid was added; the sediment was sonicated for another 20 minutes, added with 3.0 mg of polylysine powder, stirred at 4°C for 24 hours, and then centrifuged again for sediment collection; it was added with appropriate amount of sterile water for ultrasonic dispersion for around 2 hours and then autoclaved to sterilize for later use.

### 2.2. Property Characterization of Silicon Nanoparticle and Its Impact on Cell Viability

The PLL-modified silicon nanoparticles were prepared into 1 mg/mL suspension, and the particle size and potential of the nanoparticles were analyzed with a laser particle size potentiometer. At the same time, the optical microscope and transmission microscope were utilized to observe its morphology. The cell survival rate was detected by MTT method, and the specific operation method was as follows. CRC cell lines HT29 and SW480 were inoculated at 5 × 10^3^ cell/well into 96-well plates, added with different concentrations of PLL-modified silicon nanosuspension (10, 20, 30, 40, 50, 60, 70, 80, 90, and 100 *μ*g/mL) prepared with Dulbecco's modified Eagle medium (DMEM); the liposome transfection reagent (Invitrogen Lipofectamine ™ 2000) was used as a control; after 24 hours of incubation, 100 *μ*L of 0.5 mg/mL MTT solution was added to each well to cultivate for 4 hours, and 100 *μ*L of dimethylsulfoxide (DMSO) was added to each well. The OD was detected at a wavelength of 490 nm, and the cell survival rate was calculated.

### 2.3. Design and Transfection of Interference Fragments of FLOT2 Gene

According to the FLOT2 gene sequence information in Genbank and the principle of siRNA design, the siRN sequence of FLOT2 was designed. The siRNA sequence of FLOT2 was 5′-GCCuguccCuucUG-GuaaADTDT-3′, and NCBI showed no homology with other genes. Oligonucleotide fragments were synthesized in Shanghai and annealed after dilution to form double strands. The annealed double-stranded RNA fragments of FLOT2 were linked to linear plasmid Pgenesil-1 and named FLOT2-siRNA. Empty plasmid was used as a negative control (NC).

### 2.4. Cell Transfection and Transfection Efficiency Detection of FLOT2 Gene Interference Fragments

One day before transfection, the human CRC cell strain HT29 was seeded in a 6-well plate at 5 × 10^4^ cells/well, and the cell density during transfection should be guaranteed as about 90%. Before transfection, polylysine-silicon nanoparticles were dispersed in ice-water bath by ultrasonic for 20 min. Then, polylysine-silicon nanoparticles were mixed with FLOT2-siRNA and NC plasmids, respectively, at a mass ratio of 30 : 1. At 2 *μ*g plasmid per well, the suspension of 15 *μ*L polylysine-silicon nanoparticles (4 mg/mL) was mixed with 10 *μ*L FLOT2-siRNA or NC plasmids (0.218 *μ*g/L). After standing at room temperature for 40 min, the suspension was added to HT29 cells. After 5 h culture at 37°C in 5%CO_2_ incubator, the culture medium was changed to DMEM complete medium containing serum. HT29 cells without plasmid transfection were used as a blank control (CK).

Using liposome transfection method as the control, the transfection was carried out according to the instruction of Invitrogen Lipofectamine TM 2000.The specific method of liposome transfection was as follows: transfection ratio was 1 : 3 (1 *μ*g plasmid:3 *μ*L liposome) and 2 *μ*g plasmid was transferred to each well. 10 *μ*L FLOT2-siRNA plasmid was mixed with 240 *μ*L serum-free DMEM. At the same time, 6 *μ*L liposome was mixed with 244 *μ*L serum-free DMEM culture medium and the mixture was let still at room temperature for 5 min. The medium containing plasmid and the medium containing liposome were mixed evenly and then let still at room temperature for 20 min. When cells grew to 60-80%, the culture medium was removed, and the cells were rinsed with serum-free DMEM twice and then transferred to plasmid DNA/liposome complex medium to culture at 37°C, 5%CO_2_, and saturated humidity for 6 h. Subsequently, the culture medium was changed to complete medium containing 10% calf serum, followed by culture for 24 h. The transfection efficiency was observed under the fluorescence microscope.

### 2.5. RT-PCR to Detect mRNA Expression Levels of FLOT2 and EMT-Related Molecules

The total RNA of HT29 cells was extracted by TRIzol method. After the total RNA was detected by agarose gel electrophoresis, the cDNA was synthesized by reverse transcription kit (Takara Company) at 37°C for 15 min, and 85°C for 5 s in sequence. RT-PCR primer for FLOT2 gene: FLOT2-F: 5′-CCGTGGCT GTGAGCAGTT-3′, FLOT2-R: 5′- TGTCATACACGTCCTTGATGGT -3′; RT-PCR primer for MMP-2: MMP2-F: 5′- ATTCTGGAG-ATACAATGAGGT-3′, MMP2-R: 5′-TTCACGCTCTTCAGACTT-3′; RT-PCR primer for MMP-9: MMP9-F: 5′- GAAGATGCTGCTGTTCAG-3′, MMP9-R: 5′- AAAT AGGCTTTCTCTCGGTA-3′; RT-PCR primer for E-cadherin: E-cadherin-F: 5′-GACCAAGTGA CCACCTTA-3′, E-cadherin-R: 5′-AGAGCAGCAGAATCAGAAT-3′; and RT-PCR primer for vimentin: Vimentin-F: 5′-CATTGAGATTGCCACCTAC-3′, Vimentin-R: 5′-ATCGTTGATAACCTGTCCAT-3′. With *β*-actin as an internal reference, primer Actin-F of *β*-actin: 5′- AGGGGCCGGACTCGTCATACT-3′, Actin-R: 5′- GGCGGCACCACCATGTA CCCT-3′. Each sample was amplified with the above two pairs of primers, and a 20 *μ*L reaction system was established. Three replicates were performed for each reaction in the Applied Biosystems StepOne real-time fluorescence quantitative PCR instrument. Annealing temperature was 60°C, and annealing time was 30 seconds, 30 cycles. The 2^-*ΔΔ*ct^ method [16] was used to calculate the relative expression.

### 2.6. WB to Detect the Expression Levels of FLOT2 and EMT-Related Protein

After incubating in DMEM complete medium containing serum for 48 hours, the cells were collected. The total protein of liposome and HT29 cells transfected with silicon nanoparticle transfection interference plasmid were extracted, and the content of total protein extracted was determined with bicinchoninic acid (BCA). Cellular proteins were separated by sodium dodecyl sulfate polyacrylamide gel electrophoresis (SDS-PAGE), and the proteins were transferred to polyvinylidene fluoride (PVDF) membrane by wet transfer method and then sealed with 5% skimmed milk. FLOT2 and glyceraldehyde-phosphate dehydrogenase (GAPDH) antibodies diluted at a ratio of 1 : 1000 were added separately and incubated overnight at 4°C; after it was washed thoroughly with Tris-Buffered Saline Tween (TBST) for 3 times (with 10 min/time a time), horseradish peroxidase-conjugated secondary antibody was added and incubated at the room temperature for 2 h, rinsed thoroughly with TBST for another 3 times with 10 min/time each time, and then added with color developing solution for automatic exposure in development instrument. Required photos were taken and greyscale scanning was implemented. ImageJ software was used to measure the grey values of each target protein band, and the ratio of the grey value of the target protein to that of the internal reference GAPDH protein band represented the relative expression level of the target protein.

### 2.7. Experiments for Transwell Invasion and Migration

The specific operation procedures of Transwell invasion were defined as below. Under sterile conditions, the Matrigel was diluted with serum-free DMEM at a ratio of 4 : 1 to generate the membrane surface coating. 40 *μ*L of the diluted membrane surface coating was added to the upper chamber of Transwell rapidly, which should be distributed evenly on the upper compartment membrane. The cells were incubated at the 37°C for 6 h and then inoculated. Cells in the log phase were collected, the cell suspension was prepared with serum-free DMEM after digestion, and the cell concentration was adjusted to 5 × 10^4^ cells/mL. The cell suspension was poured to the upper layer of the Transwell chamber, 750 *μ*L of DMEM complete medium was added to the lower chamber of the Transwell, and then, the solution was incubated at a temperature of 37°C for 24 hours. Transwell chamber was taken out, flushed with 0.1% crystal violet lasting for 20 minutes, and rinsed with water for 3 times. Then, the photos were taken under the microscope after drying. 500 *μ*L/well of 10% acetic acid was added to dissolve the dye on the polycarbonate membrane, and the value of each hole was measured when the wavelength was 570 nm. During the operation of the Transwell migration test, the coated filter did not contain Matrigel, the rest steps were the same as the Transwell invasion test, and the OD of every well was detected at a wavelength of 570 nm.

### 2.8. CCK8 Test

The cells were collected when they grew to 70%-80% and then suspend them in 3 mL of DMEM containing 10% FBS, 100 U/mL penicillin, and streptomycin, respectively; they were added with 200 *μ*L/well cell suspension to incubate in a plate for 24, 48, and 72 h, respectively. After the CCK8 solution was mixed with DMEM containing 10% FBS, 100 U/mL penicillin, and streptomycin in a ratio of 1 : 10, respectively, 100 *μ*L of the above mixed solution was added to each well of cells, and the culture plate was placed into the incubator for another 3 hours. The OD of every well was measured with a microplate reader at 450 nm at different incubation periods.

### 2.9. Statistical Analysis

SPSS 19.0 was used for data statistics and analysis. Measurement data were indicated as mean ± standard deviation ($\bar{x}\pm s$), and counting data were indicated with percentages. The measurement data obeying the normal distribution was compared by using the *t*-test, and measurement data not obeying the normal distribution was compared using the Wilcoxon Test. *P* < 0.05 indicated statistically meaningful difference.

## 3. Results

### 3.1. Analysis on Property Characteristics of Silicon Nanoparticles

After the silicon nanoparticles synthesized by the W/O emulsification method were modified with PLL, the electron microscope revealed that they were approximately spherical silicon nanoparticles (Figure 1(a)) with the regular morphology and uniform size (Figure 1(b)). The particle size was 5-55 nm, and the APS was 30 nm (Figure 1(c)). The analysis of particle size and potential of the nanoparticles by using the laser particle size potentiometer found that the PLL-modified silicon nanoparticles had the potential of 19.65 mV, the particle size of 65.8 nm, and the dispersion coefficient of 0.103.

### 3.2. Impacts of Silicon Nanoparticles on Cell Activity

Figure 2 showed the effects of polylysine-silicon nanoparticles and liposome reagents on the HT-29 cell activity. With the increasing concentration, the effects of polylysine-silicon nanoparticles and liposome reagents on the cell activity of HT-29 cell line showed a downward trend. At the same concentration, the survival rate of polylysine-silicon nanoparticle-treated cells was significantly higher than that of liposome transfection reagent-treated cells. When the concentration of polylysine-silicon nanoparticles and liposomes ranged from 50 *μ*g/mL to 80 *μ*g/mL, the activity of cells treated by liposomes was significantly different from that of polylysine-silicon nanoparticles (*P* < 0.05). When the concentration of polylysine-silicon nanoparticles and liposome reagent was greater than 80 *μ*g/mL, the cell activity of transfection reagent was significantly different from that of polylysine-silicon nanoparticles (*P* < 0.01).

Figure 3 showed the effects of polylysine-silicon nanoparticles and liposome reagent on the SW480 cell activity. With the increasing concentration, the effect of polylysine-silicon nanoparticles and liposome reagent on the cell activity of SW480 cell line showed a downward trend. At the same concentration, the survival rate of polylysine-silicon nanoparticle-treated cells was significantly higher than that of liposome transfection reagent-treated cells. When the concentration of polylysine-silicon nanoparticles and liposomes ranged from 70 *μ*g/mL to 90 *μ*g/mL, the activity of cells treated by liposomes was significantly different from that treated by polylysine-silicon nanoparticles (*P* < 0.05). When the concentration of polylysine-silicon nanoparticles and liposomes was 100 *μ*g/mL, the cell activity treated by liposomes was significantly different from that treated by polylysine-silicon nanoparticles (*P* < 0.01).

### 3.3. Detection on Transfection Efficiency of Silicon Nanoparticles

The plasmids were transfected with liposomes and nanoparticles to compare their TEs under a fluorescence microscope (Figure 4) so as to verify the TE of silicon nanoparticles in HT29 cells. It suggested that the fluorescence of plasmid transfected with nanoparticles was remarkably more than that of liposome transfection. At the same time, the average transfection efficiency of different methods was calculated in 5 fields. It was found that the transfection efficiency of nanoparticles was 60.58 ± 2.15% and that of liposomes was 40.29 ± 1.79% (*P* < 0.05).

### 3.4. Detection on FLOT2 Gene Expression

WB was used to detect the expression level of FLOT2 gene in HT-29 cell lines transfected with liposomes and nanoparticles. As shown in Figure 5, the FLOT2 gene expression bands were significantly weaker in FLOT2-siRNA in HT-29 cell lines transfected with liposomes and nanoparticles than those in NC and CK (Figure 5(a)). In HT-29 cell lines transfected with liposomes and nanoparticles, the expression of FLOT2 protein was significantly lower than that in NC and CK groups (Figures 5(b) and 5(c)) (*P* < 0.01).

RT-PCR was further used to detect the expression level of the FLOT2 gene. As shown in Figure 6, in the HT-29 cell line transfected with liposomes and nanoparticles, the mRNA expression of FLOT2 gene was significantly lower than the NC and CK groups (*P* < 0.01).

### 3.5. Analysis on Experiment Results of Transwell Invasion

Figure 7 showed the invasion results of the NC, CK, and FLOT2-siRNA groups. The number of invaded cells in the FLOT2-siRNA group was significantly less than that in the NC group and CK group (Figure 7(a)), and the OD value of FLOT2-siRNA group was significantly lower than that of the NC group and CK group, with significant differences (*P* < 0.01).

### 3.6. Analysis on Experiment Results of Transwell Migration

Figure 8 showed the migration results of the NC, CK, and FLOT2-siRNA groups. The number of migration cells in the FLOT2-siRNA group was significantly less than that in the NC group and CK group (Figure 8(a)), and the OD value of FLOT2-siRNA migration cells was significantly lower than that of NC group and CK group, with significant differences (*P* < 0.01).

### 3.7. Analysis on CCK8 Experiment Results

The results of the CCK8 experiment were shown in Figure 9. It suggested that the ODs of cells in NC and FLOT2-siRNA had rising trends over time, and the ODs in two groups were not statistically different at the 0^th^ and 24^th^ hour (*P* > 0.05). Starting from the 48^th^ hour, the ODs of cells in the two groups increased rapidly with time. The OD in FLOT2-siRNA was lower than that in NC at the 48^th^, 72^nd^, and 90^th^ hour, and the two had extremely observable difference (*P* < 0.01).

### 3.8. Expression of EMT-Related Genes in Different Groups

The mRNA levels of EMT-related genes, namely, MMP9, MMP2, E-cadherin, and vimentin, in different groups were analyzed. As shown in Figure 10, there was no statistical difference in the expression levels of MMP9 gene in the NC group, CK group, and FLOT2-siRNA group (*P* > 0.05). The mRNA levels of MMP2 and vimentin in the FLOT2-siRNA group were significantly lower than those in the NC group and CK group (*P* < 0.01). The mRNA level of E-cadherin in the FLOT2-siRNA group was significantly higher than that in the NC group and CK group, with significant differences (*P* < 0.01).

Figure 11 showed the expression levels of EMT-related gene protein in different groups. There was no statistical difference in the expression levels of MMP9 protein in the NC group, CK group, and FLOT2-siRNA group (*P* > 0.05). The protein expression levels of MMP2 and vimentin in the FLOT2-siRNA group were significantly lower than those in the NC group and CK group (*P* < 0.01). The expression of E-cadherin protein in the FLOT2-siRNA group was significantly higher than that in the NC group and CK group, with significant differences (*P* < 0.01).

## 4. Discussion

As a targeted technology, RNA interference technology plays a critical role in gene function verification, research on the pathogenesis of immune diseases, and prevention and treatment of infectious diseases. However, the current transfection systems commonly used in RNA interference technology have certain defects [17]. Therefore, seeking gene carriers with high TE, simple preparation, low price, and no toxicity is of important research significance. The development of nanotechnology provides a new opportunity for the application of RNA interference technology. Current studies have found that silicon nanoparticles have a better cell uptake effect. They can adhere to the cell surface and enter the cell after binding with the target gene. They are relatively less toxic to cells. Nanoparticles can also protect foreign DNA fragments from degradation of DNA enzymes in the body [18, 19]. In this study, nonylphenol polyoxyethylene ether was undertaken as a surfactant to prepare the silicon nanoparticles by the emulsification method, the nanoparticles were modified with PLL, and their properties were analyzed. The results showed that the nanoparticles had regular morphology and uniform size under an electron microscope, with an APS of 30 nm, a potential of 19.65 mV, a particle size of 65.8 nm, and a dispersion coefficient of 0.103. Appropriate surfactants were generally adsorbed on the surface of the particles, which could protect the stability of the particles to a certain extent [20]. Studies have pointed out that the smaller the nanoparticle, the greater the density of modified substance bound per unit area [21]. Moreover, the PLL used in this study was positively charged, and the surface had a large amount of positive charges after modifying the silicon nanoparticles, which enhanced the binding capacity of plasmid DNA. To verify the effect of silicon nanoparticles prepared in this article on cell activity, differences between the two groups were compared by taking liposome transfection reagent as a control. It was found that the cell survival rate of silicon nanoparticles was observably higher than that of the liposome transfection reagent at the same concentration. It indicated that the toxicity of silicon nanoparticles to cells was greatly lower than that of liposome transfection reagents. A large number of research results have shown that cationic liposome transfection reagent as a nonviral carrier has poor stability and cytotoxicity [22]. Moreover, the results of this study found that TE of the nanoparticle and liposome was 60% and 40%, respectively, which were much different from each other. The above results indicated that the silicon nanoparticles prepared had the characteristics of low impact on cell activity and high TE, so they could be widely and extensively applied in the transfection of foreign genes.

FLOT2 is a member of the floating protein family and is an important lipid raft marker protein. As a signal protein, it was involved in various events such as cell proliferation, apoptosis, adhesion, cell signal transduction, and cell surface protein stability [23, 24]. FLOT2 was related to in human neuron differentiation and axon regeneration, T cell activation and its receptor complement, and the formation of lipid raft structure and endocytosis [25, 26]. In addition, a large number of research results show that FLOT2 is closely related to formation and development of tumor. It has been found that FLOT2 gene is highly expressed in various cancers, which promotes the occurrence and metastasis of tumor [27]. siRNA-mediated FLOT2 protein can greatly reduce the activity of Src tyrosine kinase and alleviate the epithelial-mesenchymal transformation process of nasopharyngeal carcinoma cell strains [14]; and siRNA-mediated FLOT2 protein can also reduce the growth and invasion of esophageal squamous cancer [28]. The results of this study found that the FLOT2 protein expression in the FLOT2-siRNA group was decreased greatly comparing with the NC group (*P* < 0.01). The mRNA level in the FLOT2 gene in the FLOT2-siRNA group was much lower than that in the NC group (*P* < 0.05), which was consistent with the current research results. This article further studied the impacts of the FLOT2 gene on the invasion and metastasis ability of CRC cells and found that the ODs of invasion cells and migration cells in NC were ncreased greatly in contrast to the FLOT2-siRNA with *P* < 0.01 and *P* < 0.05, respectively. The OD in both groups increased with time. The OD of cells in FLOT2-siRNA cells was lower than that in NC at the 48^th^, 72^nd^, and 96^th^ hour (*P* < 0.001). Wang et al. [29] applied RNA interference technology to downregulate the expression of FLOT2 and found that the proliferation, invasion, and migration of gastric cancer cells were inhibited effectively, which was similar to the results of this article.

MMPs have been proved to be the most important proteolytic enzyme affecting matrix degradation during EMT [30]. Type IV gelatinase MMP-2 and MMP-9 are the most important MMPs [31]. Many studies have reported the role of MMP-2 and MMP-9 in the process of EMT [32, 33]. The results of this study showed that there was no statistical difference in mRNA level and protein expression of MMP9 gene in the NC group, CK group, and FLOT2-siRNA group (*P* > 0.05), and the mRNA level and protein level of MMP2 in the FLOT2-siRNA group were significantly lower than those in the NC group and CK group (*P* < 0.01). It was noted that siRNA-mediated FLOT2 protein downregulates the expression of MMP-2 and degrades the extracellular matrix in CRC cells, thus playing an important role in the EMT process of CRC cells. In addition, E-cadherin and vimentin are considered the most important epithelial cell markers and mesenchymal cell phenotypic markers during EMT [34]. Many experiments have confirmed that the decrease of E-cadherin protein activity is the first step for tumor cells to acquire the ability of dedifferentiation and invasion [35], that is, E-cadherin protein can inhibit the invasion and migration of tumor cells [36]. Meanwhile, overexpression of vimentin can promote the invasion and migration of tumor cells [37], while blocking its expression through molecular biological methods can significantly reduce the invasion ability of tumor cells. The results showed that the mRNA level and protein expression of vimentin in the FLOT2-siRNA group were significantly lower than those in the NC group and CK group (*P* < 0.01) and that the mRNA level and protein expression of E-cadherin in the FLOT2-siRNA group were significantly higher than those in the NC group and CK group (*P* < 0.01). These results suggest that siRNA-mediated FLOT2 protein may play an important role in EMT by downregulating vimentin expression and upregulating E-cadherin expression in CRC cells. Above, this study confirmed that FLOT2 inhibits the migration and invasion of CRC cells by regulating the expression levels of MMP-2, E-cadherin, and vimentin during EMT.

## 5. Conclusion

Based on nanotechnology, the silicon nanoparticles were modified and applied to the construction of RNA interference plasmids. The TE of nanoparticles on the interference plasmids and their effects on cell viability were discussed. The FLOT2 gene in invasion, migration, and proliferation of CRC cell was further studied. However, there are still some shortcomings in this article. This article only studied the TE based on the FLOT2 gene fragment and did not use genes of different fragment sizes for the study. Therefore, it is unclear whether the TE of silicon nanoparticles will be affected by the gene fragment size. In the future, different fragment sizes will be added to explore whether the TE of silicon nanoparticles is related to the size of gene fragments. In the study, an RNA interference plasmid with high transfection efficiency and low cytotoxicity was established based on nanotechnology. It was found that siRNA-mediated FLOT2 protein inhibits the invasion, migration, and proliferation of CRC cells by regulating the expression of EMT-related genes, which provides a scientific basis for clinical treatment of CRC.

## Figures and Tables

**Figure 1:** Analysis on property characteristics of silicon nanoparticles. (a, b) The morphology of silicon nanoparticles under transmission microscope and optical microscope, respectively. (c) The range of particle size.

**Figure 2:** Effect of silicon nanoparticles on cell viability of HT29 cells. (^∗^*P* < 0.05 indicates a statistical difference compared with liposome-transfected cells; ^∗∗^*P* < 0.01 indicates a significant difference compared with liposome-transfected cells).

**Figure 3:** Effect of silicon nanoparticles on SW480 cell activity (^∗^*P* < 0.05 indicates a statistical difference compared with liposome-transfected cells; ^∗∗^*P* < 0.01 indicates a significant difference compared with liposome-transfected cells).

**Figure 4:** Fluorescence images of plasmid transfected with nanoparticles and liposome. (a, b) The fluorescence images of plasmid HT29 transfected with liposome and nanoparticles, respectively. (c) The fluorescence image of not transfected plasmid HT29. (d) The transfection efficiency of the two transfection methods (^∗^*P* < 0.05 indicates a statistical difference compared with liposome-transfected cells).

**Figure 5:** FLOT2 gene expression detected by WB. (a) WB development of HT-29 cells transfected with FLOT2-siRNA. (b) FLOT2 protein expression in HT-29 cells transfected with liposomes. (c) FLOT2 protein expression in HT-29 cells transfected with nanoparticles (^∗∗^*P* < 0.01 indicates an extremely significant difference compared with the NC group).

**Figure 6:** Comparison in mRNA level of FLOT2 gene. (a) FLOT2 mRNA level in HT-29 cells transfected with liposome plasmid. (b) FLOT2 gene mRNA level in HT-29 cells transfected with nanoparticles. (^∗∗^*P* < 0.01 indicates an extremely significant difference compared with the NC group).

**Figure 7:** Experiment results of Transwell invasion in different groups. (a) The images of Transwell invasion in two groups. (b) The comparison in ODs of Transwell invasion in two groups.

**Figure 8:** Analysis on experiment results of Transwell migration in different groups (a) The images of Transwell migration of cells in each group (b) The ODs of Transwell migration in each group. Note: ^∗∗^*P* < 0.01 suggested the difference with the NC group was extremely obvious.

**Figure 9:** Comparison in CCK8 experiment results of different groups Note: ^∗∗^*P* < 0.01 suggests extremely obvious differences versus NC group, and ^∗^*P* < 0.05 represents a statistical difference compared with the NC group.

**Figure 10:** Expression levels of EMT-related genes in different groups. ^∗∗^*P* < 0.01 represents significant differences compared with NC group.

**Figure 11:** EMT-related protein expression levels in different groups. (a) Developed images of EMT-related protein in different groups. (b) EMT-related protein expression levels in different groups (^∗∗^*P* < 0.01 represents extremely obvious differences versus the NC group).

## Data Availability

All data, models, and code generated or used during the study appear in the submitted paper.
